# Thermodynamics of Cadmium Sorption on Different Soils of West Bengal, India

**DOI:** 10.1155/2014/216451

**Published:** 2014-02-06

**Authors:** Tanmoy Karak, Ranjit Kumar Paul, D. K. Das, Romesh K. Boruah, Indira Sonar

**Affiliations:** ^1^Department of Agricultural Chemistry and Soil Science, Faculty of Agriculture, Bidhan Chandra Krishi Viswavidyalaya, Mohanpur, Nadia, West Bengal 741252, India; ^2^Upper Assam Advisory Centre, Tea Research Association, Dikom, Assam 786101, India; ^3^Division of Statistical Genetics, Indian Agricultural Statistics Research Institute, New Delhi 110012, India

## Abstract

A sorption study was conducted on different soils collected from five agroecological zones of West Bengal, India, to understand the soil environmental behavior and fate of cadmium. For this purpose batch adsorption experiments were carried out at the native soil pH and at three different temperatures (25°C, 35°C, and 45°C). The adsorption data fitted by a linear least squares technique to the different sorption isotherms. Most data obtained give the good fit to both Freundlich and modified Langmuir isotherms, but they are not consistent with the linear Langmuir adsorption model. Thermodynamic parameters, namely, thermodynamics equilibrium constant at a particular temperature T  (*K*_*T*_^0^), Gibbs free energy at a particular temperature T  (Δ*G*_*T*_^0^), and change of enthalpy (Δ*H* ^0^) and change of entropy at temperature T  (Δ*S*_*T*_^0^), were also determined by applying sorption value and concentrations of Cd in equilibrium solution within the temperature range. The thermodynamic parameters revealed that Cd sorption increases as the values of *K*_*T*_^0^, Δ*G*_*T*_^0^, Δ*H* ^0^, and Δ*S*_*T*_^0^ were increased on reaction temperatures. The spontaneous sorption reaction can be concluded due to high values of Δ*G*_*T*_^0^. The positive values of Δ*H* ^0^ indicated that the Cd sorption is an endothermic one. Under these present conditions, the soil and its components possibly supply a number of sites having different adsorption energies for cadmium sorption.

## 1. Introduction

Contamination of heavy metals in soils is increasingly concerned in the last 6 decades [1–3]. In particular, cadmium (Cd) is one of the most important toxic metals because of its rapid increase in soil environment [4], microbially or chemically undergraded characters, and easy uptake by plants and animals [5, 6], subsequently resulting in high ecological risk. An understanding of Cd sorption process and transport pathway is thus crucial for the assessment of Cd metal contamination in soil and reclamation of such polluted soils [7]. The sorption of Cd depends on soil characters and its component such as Al-oxides, Fe-oxides, goethite, organic matter, and other chemicals and mineralogical characteristics [2, 8–10]. Despite their significant influences, temperature changes can exert an important action in regulating sorption-desorption equilibrium and bioavailability of Cd in soils. The sorption of heavy metals by soils has been extensively studied [10–12]. Results suggest that sorption appears to be a multi-step process involving an initial fast adsorption followed by a slow adsorption and diffusion into solid particles. The sorption of Cd into soil can be well described by a Freundlich or linear isotherm, whereas the closeness of Langmuir isotherm to the experimental results is lower [13–15]. Estimation of the effect of individual components on the sorption of cadmium in soils can be drawn from different sorption isotherms.

The effect of temperature on Cd sorption at soil-water interface was also extensively studied [2, 16, 17]. Their results suggest that sorption of Cd in soil is favored at higher temperature. The equilibrium constant for the reaction at a particular reaction temperature (*T*), *K*_*T*_^0^, is related to the free energy change by Δ*G*_*T*_^0^ = −*RT*ln⁡*K*_*T*_^0^. Since *K*_*T*_^0^ increases with temperature in endothermic reactions, the formation of reaction products will be favored at high temperature. Therefore, a thermodynamic change in a reaction is more important to predict the reaction properties and direction of a reaction. Quantification of free energy changes (Δ*G*_*T*_^0^) at a particular temperature (*T*) is also directly related to the transport of solute element from bulk solution into the appropriate site of the double layer or clay minerals lattice. It is also helpful to understand the sorption processes. Sposito investigated that thermodynamics approach can predict the sorption of metal from an initial nonequilibrium state to final state [18].

In view of the above, the present study was undertaken to understand the sorption behavior of Cd using conventional Langmuir, modified Langmuir, and Freundlich equations and to determine thermodynamic and sorption parameters for different soils collected from five agroecological zones of West Bengal, India.

## 2. Materials and Methods

Five soil samples with contrasting soil properties were collected from the A1 horizons of five agroecological zones in West Bengal, India (Figure 1).

The agroecological zones were Lakhsmikantapur series (Sample ID: S_1_), Kakdwip series (Sample ID: S_2_), Diamond harbor series (Sample ID: S_3_), Chondrokona series (Sample ID: S_4_), and Bohorasol series (Sample ID: S_5_). The collected soils were air dried, sieved (<2 mm), and stored at room temperature in polyethylene bags. Twenty samples of each kind of soil were analyzed for physicochemical properties (Table 1). The pH and electrical conductivity of the samples were determined in saturated paste extracts [19]. The soil pH was carried out on soil slurries having soil : water ratios as 1 : 2.5 using a pH meter (Systronics India Ltd., model 239) and electrical conductivity (EC) was determined on soil slurries having soil : water ratios as 1 : 5 with a conductivity meter (Systronics India Ltd., model 507). Organic carbon and particle size distribution were analyzed by the Walkley-Black method [19] and the international pipette method [20], respectively. CaCO_3_ was estimated by standard analytical methods as described by Page [21]. 0.005 M DTPA solutions were used to extract the available pool of cadmium, following the method as described by Lindsay and Norvell [22]. Briefly, 10 mL of 0.005 M diethylene triamine pentaacetic acid (DTPA), 0.1 M triethanolamine (TEA), and 0.01 M CaCl_2_ solution (pH = 7.3) were added to 5 g of soil and the sample was shaken for 2 h. After centrifugation (4000 rpm for 10 min) the supernatant was filtered through 0.2 *μ*m Whatman filter paper in a 25 mL polycarbonate volumetric flask and diluted to 25 mL with deionized water.

For Cd sorption studies, 2 g soil sample (triplicate) was placed in 50 mL screw-capped polypropylene air tight centrifuge tube with 20 mL 0.025 N NaCl solution having 5, 10, 15, 20, 25, 30, 35, 40, 50, 60, 75, and 100 mg Cd L^−1^ (final Cd concentrations). The centrifuge tubes were placed in temperature controlled orbital shaker to study the effect of reaction temperature at 25°C, 35°C, and 45°C. The equilibrium time for reaction was 25 hours. Original soil pH was maintained by addition of dilute NaOH or HCl. To prevent the thin water layer on the soil colloid surface, the soil suspension was shaken every half an hour. At the end of reaction, the samples were centrifuged at 2500 ×g for 5 minutes. Solution was filtered using 0.2 *μ*m Millipore filter paper and filtrate was stored at 4°C. To prevent any microbial growth in filtrate, 2 drops of chloroform were added. After completion of all experiment the equilibrium concentrations (*C*_*e*_), as well as total and DTPA extractable Cd, were determined using atomic absorption spectrophotometer, model Varian Spectra 250 plus. The soil solid-phase Cd was calculated from the difference between initial Cd concentrations (*C*_*i*_) and those in solutions after equilibration. Statgraphics and computations and illustrations were made by using Statgraphics and Excel packages.

### 2.1. Evaluation of Sorption Data

The Langmuir and Freundlich equations are based on the kinetic theory of gases and are extensively used to describe gas adsorption on solids [23]. These equations are often applied to the adsorption of liquids and ions from solutions by solids.

The Langmuir adsorption equation can be written as

(1) $$\begin{array}{c} \frac{x}{m}=\frac{kbC_{e}}{\left(1+kC_{e}\right)}, \end{array}$$

where *x*/*m* = amount of Cd adsorbed per unit weight of soil [mg kg^−1^], *k* = a constant related to the binding energy [dm^3^ mg^−1^], *b* = adsorption maxima [mg kg^−1^], and *C*_*e*_ = equilibrium Cd concentration in soil solution [mg dm^−3^]. Equation (1) can be rearranged to give

(2) $$\begin{array}{c} \frac{C_{e}}{\left(x/m\right)}=\left(\frac{1}{kb}\right)+\left(\frac{C_{e}}{b}\right). \end{array}$$

Equation (2) is hereafter refered to as conventional Langmuir equation. A plot of *C*_*e*_/(*x*/*m*) versus *C*_*e*_ gives a straight line from which *b* (gradient^−1^) and *k* (gradient/intercept) can be obtained.

The amount of Cd adsorbed by the soils was calculated using

(3) $$\begin{array}{c} \left(\frac{x}{m}\right)=\frac{\left\{\left(C_{i}-C_{e}\right)/V\right\}}{W}+\text{CV}, \end{array}$$

where *C*_*i*_ is the initial Cd concentration (mg·dm^−3^), *V* is the volume of the initial solution, dm^3^, *W* is the weight of a soil sample, kg, and CV is the correction value (amount of Cd extracted by DTPA) (mg·kg^−1^); Freundlich equation can be written as follows:

(4) $$\begin{array}{c} \log\left(\frac{x}{m}\right)=\log K_{f}+\left(\frac{1}{n}\right)\log C_{e}, \end{array}$$

where *K*_*f*_ and 1/*n* denote the empirical Freundlich constant.

### 2.2. Thermodynamic Consideration of Sorption Reaction

The procedure outlined by Biggar and Cheung [24] was followed to calculate thermodynamics equilibrium constant at reaction temperature *T* (absolute scale), *K*_*T*_^0^ and it can be formulated as

(5) $$\begin{array}{c} K_{T}^{0}=\left(\frac{a_{s}}{a_{e}}\right)=\left(\frac{\lambda_{S}C_{S}}{\lambda_{e}C_{e}}\right), \end{array}$$

where *a*_*s*_ = activity of adsorbed metal on soils at temperature *T*, *a*_*e*_ = activity of metal in soil solution at equilibrium state at temperature *T*, *γ*_*s*_ = activity coefficient of sorbed metal in soils at temperature *T*, *γ*_*e*_ = activity coefficient of sorbed metal in solution at temperature *T*, *C*_*s*_ = m metal adsorbed per L of solution in contact with the soil surface at temperature *T*, *C*_*e*_ = Mm metal per L of solution at equilibrium in contact with the soil surface at temperature *T*.

At low concentrations, the activity coefficient approaches to the unity and (5) can be written as follows [7]:

(6) $$\begin{array}{c} K_{T}^{0}=\frac{C_{s}}{C_{e}}. \end{array}$$

The values of *K*_*T*_^0^ were obtained by plotting *C*_*s*_ versus *C*_*e*_ and extrapolating to zero *C*_*s*_.

The standard Gibbs free energy at a particular temperature *T*, Δ*G*_*T*_^0^, was calculated as follows:

(7) $$\begin{array}{c} \Delta G_{T}^{0}=-RT\ln K_{T}^{0}. \end{array}$$

The change of enthalpy Δ*H* ^0^ with change of reaction temperature range from *T*_*i*_ to *T*_*f*_ can be expressed as vant Hoff isochore (7)

(8) $$\begin{array}{c} \;\frac{d\left(\ln K_{T}^{0}\right)}{dT}=\frac{\Delta H^{0}}{RT^{2}}. \end{array}$$

On integration within limit *K*_*i*_^0^ and *K*_*f*_^0^ with respective temperature range from *T*_*i*_ to *T*_*f*_ can be obtained

(9) $$\begin{array}{c} \int_{K_{i}^{0}}^{K_{f}^{0}}d\ln K=\left(\frac{\Delta H^{0}}{R}\right)\int_{T_{i}}^{T_{f}}T^{-2}dT. \end{array}$$

Therefore,

(10) $$\begin{array}{c} \Delta H^{0}=\left(\frac{RT_{i}T_{f}}{\left(T_{f}-T_{i}\right)}\right)\ln\left(\frac{K_{f}^{0}}{K_{i}^{0}}\right), \end{array}$$

where *K*_*f*_^0^ and *K*_*i*_^0^ are thermodynamics equilibrium constants at temperatures *T*_*f*_ and *T*_*i*_, respectively, where *T*_*f*_ > *T*_*i*_ and *R* is universal gas constant.

Determination of reaction enthalpy Δ*H* ^0^ can be calculated from vant Hoff plot by ln⁡*K* versus 1/*T*.

The change of entropy at temperature *T*, Δ*S*_*T*_^0^, was calculated from the following:

(11) $$\begin{array}{c} \Delta S_{T}^{0}=\frac{\left(\Delta H^{0}-\Delta G_{{\;}^{T}}^{0}\right)}{T}. \end{array}$$

## 3. Results and Discussion

Soil samples used in the study differed significantly in their physical and chemical properties (Table 1). Cation exchange capacity (CEC) varied from 6.14 to 29.87 (cmol (p^+^) kg^−1^) with soils, representing mostly acidic to basic reaction. The physical chemical properties show that S_1_, S_2_, and S_3_ are alkaline in nature, whereas S_4_ and S_5_ are acidic in nature.

The five soil samples varied appreciably in their ability to sorb added cadmium in soil solution irrespective of initial Cd concentrations affected by reaction temperatures (Figure 2).

The sorption ability increases with rise in temperature. In all experimental soils the sorption was appreciable and changes at high reaction temperature, that is, 45°C. The highest Cd (9.14%) was adsorbed by soil S_3_ at 45°C, whereas this value was only 2.6% for S_5_ at the same temperature at *C*_*i*_ of 100 mg L^−1^. These values were 6.9 and 1.8% for soils S_3_ and S_5_ at 25°C, whereas these values were 7.9 and 2.1% at 35°C, respectively. Percent adsorption was more pronounced at low *C*_*i*_. Soil, S_3_, has more sorption capacity versus the other soils. Sorption capacity follows the sequence S_3_ > S_2_ > S_1_ > S_4_ > S_5_. The increasing temperature increases the sorption of Cd in soil because temperature may increase the rate of aggregation of suspended materials which may cause the adsorption in faster rate. The sorption ability of five soils increased with increase in clay content, pH, and calcium carbonate percentage. The increased sorbed capacity of soil with presence of increased amount of clay may be due to high charge density of both the planer [25] and edge sites [26]. On the other hand this high charge density leads to a greater dehydration to fasten Cd^2+^ ion mobility from soil solution to soil [27]. Sorption of Cd with increase in soil pH also plays a crucial role because it directly controls the solubility of cadmium hydroxides as well as its carbonates and phosphates [28]. Sorption of Cd was more at high pH. This is because of less competition from H_3_O^+^ ions compared to soils having low pH [29]. Reed et al. [30] also reported similar observations. The increase of Cd sorption with increasing soil pH increases Cd^2+^ retention of soil surface via adsorption, inner sphere surface complexation, and/or precipitation and multinuclear type reactions [31]. Cadmium (II) is a closed shell cation having complete valence orbital (5d^10^) which favors columbic type attraction at soil surface for sorption as opposed to inner sphere surface reactions through sharing of electrons [32] and which also may contribute to our findings. CEC also affect sorption of Cd. Among these soils, the one having low CEC sorbed much less Cd than that having high CEC. Singh et al. [33] also observed that CEC plays an important role in the sorption of Cd in soils.

Every 10°C increase in temperature, percentage Cd sorption increases 5.8 to 6.19% for S_1_, 6 to 6.9% for S_2_, 7.6 to 11.11% for S_3_, 3.8 to 5.0% for S_4_, and 1.8 to 2.6% for S_5_ from higher to lower concentration of added Cd. The increase in sorption with rise in temperature indicates that Cd sorption is exothermic in nature (see later in thermodynamic approach). The marked effect of Cd sorption with temperature was found in acidic soils (S_4_ and S_5_) versus alkaline soils (S_1_, S_2_, and S_3_). The results from this study corroborated with those reported by Almås et al. [16]. Increasing temperature enhances the rate of metal reaction with soil constituents [16] and this effect has been ascribed to a diffusion-controlled metal penetration in the mineral structure [34]. The general explanation can also be recognized from our experiment on the adsorption of Cd in soil that increases with temperature due to the decrease in the activation energy of sorption reaction which promotes the sorption kinetics.

Cadmium sorption on soils also depends on the presence of organic carbon in soils. The sorption of Cd by different soils decreases with increase in organic carbon. This may be due to the formation of stable soluble metal-organic complex with soil organic matter facilitating the persistence of Cd in soil solution [35]. The increased temperature may also have facilitated the biological degradation of organic materials, which may be the possible reason of the observed fact.

### 3.1. Modeling of Sorption Data

For all experimental soils, sorption data of Cd was initially tried to be fitted in conventional Langmuir equation (2) to predict the behavior of Cd sorption in soils (Table 2). The values of sorption maxima (*b*) ranged from 24.39 to 99.01 mg kg^−1^. In all cases, a sorption maximum (*b*) was increased with rise in temperature. Percent increase of *b* from 25°C to 35°C and 35°C to 45°C was 6.26 and 10.89 for soil S_1_, 13.97 and 14.12 for S_2_, 12.46 and 16.22 for soil S_3_, 3.57 and 18.18 for S_4_, and 7.05 and 9.42 for S_5_ soil. Sorption was maximum for soil S_3_ due to higher clay content. Bolton and Evans [36] also reported that clay content in soil was significantly correlated to sorption maximum. Pronounced change of *b* in soil S_4_ may be due to more dissolution of organic acids present in soil and the more competition between H^+^ and Cd^2+^ contributes to the observed fact. Results from this experiment bear similarities to those reported by Bruemmer et al. [37]. They also found that the adsorption of Cd on soil increases with increase of sorption reaction temperature.

The affinity of metal bonding varied with soil types and sorption temperature. Bonding energy (*k*) increases with increase in temperature and ranges from 0.018 to 0.055 L mg^−1^. The results are very much similar to those reported by Adhikari and Singh [7]. Increasing *k* with rise in temperature not only indicates the increased sorption but also indicates that at higher temperature sorption of Cd in soil may shift from physisorption to chemisorptions [31].

The Langmuir one-site isotherm is conceptually valid for monolayer sorption on a surface containing a finite number of binding sites. Moreover, the treatment assumes uniform energies of sorption on the surface and no transmigration of adsorbates into the plane of the surface. Such restrictions are not applicable to solids characterized by heterogeneous adsorptive surface like those found in soil systems. Data analysis and interpretations solely on Langmuir adsorption maximum (*b*) should be undertaken with care since it does not outline some sorption particularities as illustrated in figures (Figures 3(a), 3(b), 3(c), 3(d), and 3(e)).

When the sorption data were plotted according to the conventional Langmuir equation (2), the frequently reported linear relationship was obtained for equilibrium concentration (*C*_*e*_) lower than 33.74, 33.35, and 33 mg L^−1^ for S_1_, 33.17, 32.64, and 31.95 mg L^−1^ for S_2_, 31.84, 31.18, and 30.15 mg L^−1^ for S_3_, 34.00, 33.80, and 33.51 mg L^−1^ for S_4_, 34.21, 34.09, and 33.83 mg L^−1^ for S_5_ at 25°C, 35°C, and 45°C, respectively (Figures 3(a), 3(b), 3(c), 3(d), and 3(e)). Above those values of *C*_*e*_ the linearity of curves follows another path. These deviations also follow the linear Langmuir relationship, which suggest that the existence in each soil with different temperature has two sites of adsorption populations. These two different sites have widely differing affinity for Cd, each of which can be described by two-site Langmuir relationship having varied *k* and *b* values. To describe this phenomenon, *C*_*e*_/(*x*/*m*) versus *C*_*e*_ curve (2) was resolved into two-site equation using modified Langmuir sorption equation described by Syers et al. [38]. Consider the following:

(12) Ce(x/m)=kIbI(Ce(1+kICe))+kIIbII(Ce(1+kIICe))  modified  Langmuir.

The values of coefficients *k*_I_ and *b*_I_ for part I curve and *k*_II_ and *b*_II_ for part II curve were calculated to know the sorption maxima and bonding energy separately using regression equations (Table 3). Modified Langmuir equation give better fit for Cd sorption (*R* ^2^ = 0.990–0.999**) than conventional Langmuir equation (*R* ^2^ = 0.784–0.875) in all ranges of sorption temperatures. Harter and Baker [39] suggested that the modified Langmuir isotherm provides better linearity rather than conventional Langmuir isotherm, because the former considers the ratio of adsorbed and desorbed cations. The adsorption maxima for part I (*b*_I_) was smaller versus part II (*b*_II_) irrespective of treatment and temperature for all the soils. Adsorption maxima for part I (*b*_I_) was found for S_3_ at 45°C (49.26 mg kg^−1^) and it was minimum for S_5_ (11.90 mg kg^−1^). At 25°C and 35°C it was 38.02 and 42.37 mg kg^−1^ for S_3_, whereas 10.49 and 10.66 mg kg^−1^ were obtained for S_5_. A highest adsorption maximum for part II (*b*_II_) was for S_3_ at 45°C (188.61 mg kg^−1^) and it was minimum for S_5_ (76.92 mg kg^−1^). At 25°C and 35°C it was 172.41 and 175.44 mg kg^−1^ for S_3_, while the same was 56.82 and 71.43 mg kg^−1^ for S_5_. The values of *b*, obtained by using modified Langmuir adsorption isotherm, follow the same trend observed in conventional Langmuir equation. Cadmium sorption maxima for part I (*b*_I_) was five times less than that of part II (*b*_II_). This deviation may be due to the high initial concentration (*C*_*i*_) of Cd. Lower values of *b*_I_ on part I curve may be due to the less adsorption of Cd on soil surface up to *C*_*i*_ equal to 35 mg L^−1^ whereas higher values of *b*_II_ on part II curve may be due to high cadmium adsorption on soil. The ranges of *k*_I_ and *k*_II_ were 0.08 to 11.24 and 0.005 to 0.01 mg L^−1^, respectively. The high value of *k*_I_ indicate the strong bonding between Cd and soil particles prevailing chemisorption on soil surface and it mainly rises up to 35 mg L^−1^ as Cd is added in all experimental soils irrespective of reaction temperature. On other hand the lower value of *k*_II_ conforms the physisorption of Cd on soil surface along with the precipitation of Cd at high soil pHs. The values of *k*_I_ and *k*_II_ also suggest that there are at least two forms of Cd sorbed on soils. The one at low concentrations (*C*_*i*_ = 35 mg L^−1^ Cd) represents specially sorbed Cd at high energy surfaces having low dissociation constant. The other one at high metal concentrations (*C*_*i*_ > 35 mg L^−1^) may be the indicative of loosely held metal at low energy surfaces having high dissociation constant or precipitation as suggested by Adhikari and Singh [7]. Thus differences in bonding affinity for Cd among all soil types were more prominent at low level of Cd pollution.

Table 4 shows the Freundlich constants of Cd sorption isotherms of five different agroecological top soils in the pH range of 5.61–8.62. Freundlich adsorption isotherm better fits the data (*R* ^2^ = 0.901–0.981**) versus the Langmuir isotherm (*R* ^2^ = 0.791–0.875**). For all experimental soils the values of *K*_*f*_ and *n* were greater at higher temperatures. The values of *K*_*f*_ were >17.968 for S_2_ at 45°C whereas it was <1.241 for S_5_ at 25°C. All *K*_*f*_ values were >1. Another constant *n* follows the same trend like *K*_*f*_.

### 3.2. Thermodynamic Variables of Cadmium Sorption in Soils

Vant Hoff's equation (10) provides a way of measuring the enthalpy of a reaction without using calorimeter. Equilibrium compositions are measured over a range of temperature (at constant pressure), and ln⁡*K* is plotted against 1/*T*. It is revealed from (10) that the slope is −Δ*H* ^0^/*R*. On account of the temperature dependence of the reaction enthalpy, this slope depends on the temperature and so the line is not expected to be perfectly straight. In practice, however, Δ*H* ^0^ normally depends only weakly on the temperature [23]. On sorption experiments of Cd in soil, it was found that the sorption of Cd increases with temperature, and therefore according to Le Chatelier's principle, the sorption of Cd in soil is endothermic one. In order to find the reason for behavior of Cd sorption in soils we need to look for thermodynamics variables like *K*_*T*_^0^, Δ*G*_*T*_^0^, Δ*H* ^0^, and Δ*S*_*T*_^0^. The data in Table 5 indicate that values of *K*_*T*_^0^ increased with rise in temperature from 25°C to 45°C ranging from 0.021 to 0.123. Higher values of *K*_*T*_^0^ indicate the lower amount of *C*_*e*_. The variations of *K*_*T*_^0^ with respective sorption temperatures may be due to soil pHs. The changes of pH have commonly been attributed to the preferential adsorption of CdOH^+^ [40], the adsorption of Cd^+2^ [41], proton competition for adsorption sites [42], variation in the negative surface charge density of the soil [2, 43], and acid catalyzed dissolution of reactive oxide sites [13, 44] or precipitations as carbonates, hydroxides, and phosphates. In all soils, the free energy change (Δ*G*_*T*_^0^) of Cd sorption is positive and these values decrease with temperature which suggests the spontaneity of adsorption process with rise in temperature [45]. The spontaneity of sorption of Cd follows the order S_3_ > S_2_ > S_1_ > S_4_ > S_5_ and this is also the same agreement that was found in sorption isotherm.

The values of Δ*H* ^0^ of Cd sorption were found to be positive and ranging from 5.81 to 9.44 (kj mol^−1^). The positive values of Δ*H* ^0^ conform the endothermic Cd sorption process in soils and spontaneity is favored by high temperature. Δ*H* ^0^ values follow the same trend that was found in *K*_*T*_^0^.

The values of Δ*S*_*T*_^0^ were found positive at higher adsorption temperature (45°C) and negative at 25°C. For soil S_4_ and S_5_ the values of Δ*S*_*T*_^0^ were also negative. |Δ*S*_*T*_^0^| ranges from 0.01 to 1.26 j mol^−1^. The positive values of Δ*S* ^0^ with higher temperatures indicate that the sorption of Cd is also favored by high temperature, whereas negative values cannot be able to bear the spontaneity of Cd sorption at lower temperature. However, the overall system in Cd sorption seemed to be endothermic, which may be attributed to the formation of different structural type of hydrated species of Cd ion and their movement from soil solution to soil. Roth et al. [46] reported that entropies are positive (just not for CS-MO) indicating that the adsorption is irreversible. Furthermore, entropies for the all soil are of the same order range as those determined on a soil from Aspach le Bas in Eastern France (Alsace-Haut Rhin) by Roth et al. [46].

## 4. Conclusions

Sorption of Cd was facilitated by temperature. At higher temperature Cd sorption was maximum in all experimental soils. Cd sorption data can be described satisfactorily by modified two surfaces, Langmuir isotherm and Freundlich isotherm. The conventional Langmuir equation failed to describe sorption of Cd in soils. The occurrence of Cd toxicity will be less in soil having higher pH, clay content, CaCO_3_, and CEC. Acidic soils are more vulnerable to Cd toxicity; even a small initial concentration of Cd may account for problem of Cd pollution and its toxicity to plants and underground water. These results also demonstrate that increasing amount of indigenous soil organic matter may be the factor of Cd toxicity and its mobility in soils via the formation of soluble Cd-organic complexes.

On the basis of thermodynamic parameters, namely, Δ*G*, Δ*H*, and Δ*S*, of adsorption kinetics it can be concluded that Cd sorption is endothermic and irreversible. Temperature always favors the sorption process. This observed phenomenon proves that the Cd toxicity in soils of India or other tropical countries would not be a serious problem due to more sorption of Cd by soils if temperature increases. Thus soil properties and soil environment particularly temperature need to be specially emphasized to minimize Cd toxicity in India or any other tropical country.

## Figures and Tables

**Figure 1:** Location map (not in scale) of the sampling site. S_*n*_ stands for sampling location.

**Figure 2:** Amount of Cd adsorbed at equilibrium as a function of three different temperatures for the experimental soils [(a) S_1_, (b) S_2_, (c) S_3_, (d) S_4_, and (e) S_5_] at different Cd concentrations.

**Figure 3:** Isotherm for the sorption of added Cd by the soils obtained using the conventional Langmuir equation; breaks in the isotherms are indicated by arrows and line of each plot represents modified Langmuir equation. (a) S_1_, (b) S_2_, (c) S_3_, (d) S_4_, and (e) S_5_. -∘-, -*▵*-, and -*◊*- for 25, 35, and 45°C.

**Table 1:** Physicochemical properties of the five experimental soils collected from different agroecological zones of West Bengal, India (data represent mean of tree replications ± SD).

Property	Soil				
	S_1_	S_2_	S_3_	S_4_	S_5_
pH (1 : 2.5) H_2_O	7.89 ± 1.78	8.09 ± 3.27	8.62 ± 3.39	6.02 ± 1.14	5.61 ± 2.03
O.C (g kg^−1^)	7.03 ± 1.05	6.02 ± 2.19	5.21 ± 1.79	8.21 ± 1.28	8.65 ± 3.17
CEC [cmol (p^+^) kg^−1^]	22.13 ± 3.79	25.39 ± 5.01	29.87 ± 2.19	8.35 ± 2.02	6.14 ± 2.15
Clay (%)	39 ± 7.78	41 ± 8.69	48 ± 4.37	20 ± 3.92	18 ± 1.78
Sand (%)	14 ± 3.67	15 ± 2.49	18 ± 1.75	28 ± 3.15	31 ± 3.13
Silt (%)	47 ± 6.67	44 ± 4.78	34 ± 5.17	52 ± 7.53	51 ± 6.35
Texture	Silty clay loam	Silty clay	Clay	Silty loam	Silty loam
Taxonomic classification	Vertic Ustochrept	Typic Haplumbrept	Typic Paleustalf	Typic Haplumbrept	Typic Haplaquest
CaCO_3 _(%)	5.51 ± 1.49	5.62 ± 1.09	6.35 ± 1.97	0.59 ± 0.07	0.41 ± 0.12
DTPA extractable Cd (mg kg^−1^)	0.004 ± 0.001	0.006 ± 0.001	0.008 ± 0.001	0.002 ± 0.001	0.001 ± 0.001

**Table 2:** Conventional Langmuir constants of Cd sorption in soils (data represent mean of tree replications ± SD).

Sample ID	Temperature (°C)								
	25			35			45		
	Conventional Langmuir constants								
	*b* (mg kg^−1^)	*k* (L mg^−1^)	*R* ^2^	*b* (mg kg^−1^)	*k* (L mg^−1^)	*R* ^2^	*b* (mg kg^−1^)	*k* (L mg^−1^)	R^2^
S_1_	33.56 ± 4.07	0.027 ± 0.001	0.816*	37.74 ± 7.17	0.041 ± 0.001	0.828*	43.86 ± 6.19	0.045 ± 0.001	0.839*
S_2_	47.17 ± 3.85	0.029 ± 0.001	0.827*	53.76 ± 3.04	0.041 ± 0.001	0.844*	61.35 ± 7.71	0.055 ± 0.001	0.874*
S_3_	84.03 ± 7.78	0.027 ± 0.002	0.844*	89.29 ± 7.78	0.037 ± 0.001	0.860*	99.01 ± 8.79	0.045 ± 0.001	0.875*
S_4_	28.57 ± 3.79	0.022 ± 0.002	0.814*	29.59 ± 3.33	0.031 ± 0.001	0.797*	34.97 ± 6.13	0.038 ± 0.001	0.805*
S_5_	24.39 ± 3.07	0.018 ± 0.001	0.810*	26.11 ± 4.02	0.023 ± 0.001	0.784*	28.57 ± 2.07	0.034 ± 0.001	0.791*

*Significant at 0.05% level.

**Table 3:** Modified Langmuir constants of Cd sorption in soils (data represent mean of tree replications ± SD).

Sample ID	Temperature (°C)	Modified Langmuir constants					
		Part I curve			Part II curve		
		*b*_I_ (mg kg^−1^)	*k*_I_ (L mg^−1^)	*R* ^2^	*b*_II_ (mg kg^−1^)	*k*_II_ (L mg^−1^)	*R* ^2^
S_1_	25	14.26 ± 2.73	0.19 ± 0.001	0.998**	81.97 ± 5.19	0.005 ± 0.001	0.999**
	35	17.06 ± 2.97	2.08 ± 0.051	0.992**	88.50 ± 4.07	0.007 ± 0.001	0.994**
	45	20.37 ± 3.01	9.26 ± 1.93	0.991**	97.09 ± 3.79	0.008 ± 0.001	0.999**

S_2_	25	21.28 ± 3.09	0.20 ± 0.001	0.997**	111.11 ± 7.17	0.006 ± 0.001	0.992**
	35	24.75 ± 2.73	0.76 ± 0.001	0.999**	114.94 ± 7.91	0.008 ± 0.001	0.992**
	45	30.67 ± 4.07	11.24 ± 1.78	0.997**	116.28 ± 11.83	0.011 ± 0.001	0.994**

S_3_	25	38.02 ± 3.71	0.15 ± 0.001	0.999**	172.41 ± 14.07	0.007 ± 0.001	0.994**
	35	42.37 ± 5.09	0.27 ± 0.001	0.998**	175.44 ± 13.19	0.009 ± 0.001	0.999**
	45	49.26 ± 6.31	0.40 ± 0.001	0.997**	188.68 ± 11.11	0.010 ± 0.001	0.995**

S_4_	25	12.39 ± 2.07	0.12 ± 0.001	0.998**	67.57 ± 6.37	0.005 ± 0.001	0.990**
	35	12.52 ± 2.56	0.79 ± 0.003	0.998**	79.37 ± 8.19	0.005 ± 0.001	0.995**
	45	15.11 ± 1.73	4.80 ± 1.09	0.999**	90.91 ± 6.67	0.006 ± 0.001	0.996**

S_5_	25	10.49 ± 1.03	0.08 ± 0.001	0.995**	56.82 ± 7.07	0.004 ± 0.001	0.973**
	35	10.66 ± 1.11	0.16 ± 0.007	0.999**	71.43 ± 3.79	0.004 ± 0.001	0.994**
	45	11.90 ± 1.23	1.26 ± 0.001	0.999**	76.92 ± 4.09	0.005 ± 0.001	0.996**

**Significant at 1% level.

**Table 4:** Freundlich constants of Cd sorption in soils (data represent mean of tree replications ± SD).

Sample ID	Temperature (°C)	Freundlich constants		
		*K*_*f*_	*n*	*R* ^2^
S_1_	25	3.228 ± 1.17	2.298 ± 1.05	0.934**
	35	2.503 ± 1.71	3.763 ± 2.01	0.925**
	45	10.028 ± 2.13	3.824 ± 1.36	0.981**

S_2_	25	4.833 ± 1.22	2.339 ± 1.24	0.937**
	35	10.447 ± 2.19	3.419 ± 1.65	0.952**
	45	17.968 ± 3.17	4.771 ± 1.24	0.931**

S_3_	25	7.264 ± 2.13	2.145 ± 1.05	0.965**
	35	12.362 ± 1.78	2.685 ± 1.04	0.930**
	45	16.413 ± 4.01	2.899 ± 1.10	0.916**

S_4_	25	1.938 ± 0.27	1.996 ± 0.99	0.964**
	35	4.899 ± 1.11	3.171 ± 1.50	0.901**
	45	7.998 ± 2.17	4.117 ± 2.05	0.945**

S_5_	25	1.241 ± 0.01	1.808 ± 1.09	0.979**
	35	2.079 ± 0.07	2.155 ± 1.00	0.935**
	45	5.451 ± 1.78	3.588 ± 2.04	0.952**

**Significant at 1% level.

**Table 5:** Thermodynamics variables on Cd sorption at reaction temperatures on experimental soils (data represent mean of tree replications ± SD).

Sample ID	Temperature (°C)	Thermodynamics variables			
		*K*_*T*_^0^	Δ*G*_*T*_^0^ (kj mol^−1^)	Δ*H* ^0^ (kj mol^−1^)	Δ*S*_*T*_^0^ (j mol^−1^)
S_1_	25	0.034 ± 0.001	8.41 ± 1.79	8.07 ± 1.97	−1.15 ± 0.78
	35	0.044 ± 0.001	7.99 ± 1.38		0.26 ± 0.03
	45	0.053 ± 0.001	7.76 ± 1.09		0.96 ± 0.01

S_2_	25	0.049 ± 0.001	7.48 ± 1.21	7.10 ± 2.29	−1.26 ± 0.12
	35	0.063 ± 0.001	7.07 ± 1.37		0.10 ± 0.001
	45	0.079 ± 0.001	6.71 ± 1.41		1.24 ± 0.61

S_3_	25	0.087 ± 0.001	6.06 ± 1.21	5.81 ± 1.01	−0.82 ± 0.002
	35	0.104 ± 0.001	5.81 ± 1.73		0.01 ± 0.001
	45	0.123 ± 0.001	5.54 ± 1.91		0.86 ± 0.17

S_4_	25	0.026 ± 0.001	9.03 ± 1.73	8.79 ± 2.01	−0.82 ± 0.02
	35	0.032 ± 0.001	8.80 ± 1.07		−0.03 ± 0.001
	45	0.040 ± 0.001	8.50 ± 1.39		0.90 ± 0.001

S_5_	25	0.021 ± 0.001	9.63 ± 2.12	9.44 ± 1.07	−0.63 ± 0.001
	35	0.024 ± 0.001	9.51 ± 1.01		−0.21 ± 0.001
	45	0.031 ± 0.001	9.16 ± 2.09		0.89 ± 0.03
